The article "Presentation of a Segmentation Method for a Diabetic Retinopathy Patient's Fundus Region Detection Using a Convolutional Neural Network" was published in 2021. Journal: Comput Intell Neurosci.

# Presentation of a Segmentation Method for a Diabetic Retinopathy Patient's Fundus Region Detection Using a Convolutional Neural Network

**DOI:** 10.1155/2021/7714351

**Published:** 2021-07-26

**Authors:** Amin Valizadeh, Saeid Jafarzadeh Ghoushchi, Ramin Ranjbarzadeh, Yaghoub Pourasad

**Affiliations:** ^1^Department of Mechanical Engineering, Ferdowsi University of Mashhad, Mashhad, Iran; ^2^Department of Industrial Engineering, Urmia University of Technology (UUT), P.O. Box 57166-419, Urmia, Iran; ^3^Department of Telecommunications Engineering, Faculty of Engineering, University of Guilan, Rasht, Iran; ^4^Department of Electrical Engineering, Urmia University of Technology (UUT), P.O. Box 57166-419, Urmia, Iran

## Abstract

Diabetic retinopathy is characteristic of a local distribution that involves early-stage risk factors and can forecast the evolution of the illness or morphological lesions related to the abnormality of retinal blood flows. Regional variations in retinal blood flow and modulation of retinal capillary width in the macular area and the retinal environment are also linked to the course of diabetic retinopathy. Despite the fact that diabetic retinopathy is frequent nowadays, it is hard to avoid. An ophthalmologist generally determines the seriousness of the retinopathy of the eye by directly examining color photos and evaluating them by visually inspecting the fundus. It is an expensive process because of the vast number of diabetic patients around the globe. We used the IDRiD data set that contains both typical diabetic retinopathic lesions and normal retinal structures. We provided a CNN architecture for the detection of the target region of 80 patients' fundus imagery. Results demonstrate that the approach described here can nearly detect 83.84% of target locations. This result can potentially be utilized to monitor and regulate patients.

## 1. Introduction

The most prevalent cause of vision loss in people with diabetes is diabetic retinopathy; however, additional causes of harm include various eye disorders in the retinal and nonretinal visions including glaucoma, macular degeneration associated with age, and neuropathy in the vascular and cataract vision. The intensity and severity of diabetic retinopathy are often diagnosed by visual examination of the fundus by direct inspection and analyzing color pictures by an ophthalmologist. This technique is costly and time-demanding, given the enormous number of diabetes patients globally [1]. The severity of diabetic retinopathy and the diagnosis of primary illnesses are both relatively subjective, with agreement amongst qualified professionals documented variably in prior research [2, 3]. Furthermore, 75% of diabetic retinopathy patients reside in poor areas with a lack of experts and diagnostic infrastructure [4]. To prevent the development of avoidable eye illnesses, global area-based prediction systems have been established; however, large-scale diabetic retinopathy exists for such systems to detect and cure retinopathy successfully on an individual basis. As a consequence, millions of people throughout the world continue to experience vision loss due to a lack of effective diagnosis and eye care.

Automated techniques for identifying retinal disease utilizing stained fundus pictures have been developed to solve the inadequacies of conventional diagnostic approaches [5]. Decentralized technicians may check numerous patients objectively and without relying on physicians using such a gadget, reducing the burden of qualified specialists. Previous techniques to the automated detection of diabetic retinopathy, on the other hand, have substantial disadvantages that impede widespread use. Since the majority of these methods are based on short data sets of around 500 pictures in specific clinical situations, they try to diagnose large-scale diabetic retinopathy in real-world heterogeneous fundus data sets [6]. Techniques generated from certain data sets may not be applicable to fundus pictures (gained from other clinical researches and employing various types of fundus cameras, eye-opening methods, or both). Furthermore, many of these algorithms for diagnosing diabetic retinopathy depend on the manual extraction of features, which seeks to explain the prediction of anatomical structures in the fundus, such as the optic disc or blood vessels, using accurate manual characteristics. Though these manually tuned features may be applied to individual fundus data sets, they are still used to detect diabetic retinopathy using fundus photos of people who meet the prototype's demographics [7]. Although general objective features, such as acceleration of feature detection and orientation gradient histogram, have been examined as a nonspecific technique for characterizing diabetic retinopathy, these methods do not tackle weaker and disproportionate features that can be found in diabetic retinopathy. It does not go into detail on small changes in retinopathy severity [8].

Researchers have paid a lot of consideration to artificial-intelligence-based approaches in recent times, and they have been able to produce good outcomes in a variety of areas, particularly in the field of computer vision, and in some situations, they have even been able to compete with humans [9]. The preparation of specialized characteristics is another significant aspect in this domain. What has been typical in prior computer vision systems is that researchers first do extensive study to uncover certain characteristics in the input and then utilize these characteristics to execute their intended processing operations. The procedure of developing these characteristics is time-consuming and does not always provide satisfactory outcomes. The features are automatically found through artificial intelligence and data mining technologies, and then the required action is done utilizing these features. This approach offers a high level of accuracy, which is why so much study is being done in this area. As a result, in order to take advantage of the strong capabilities that these approaches give researchers in addressing artificial intelligence challenges, it is vital to get more familiar with them and address them in order to tackle their difficulties in departments [10]. In diabetic patients with diabetic retinopathy, the regular growth-based prognosis is a crucial and critical element of patient therapy. The cost of therapy is heavily influenced by the accuracy and timeliness of this care [11]. If discovered early, compensatory therapy for diabetic retinopathy is available, and it is a vital step. The weighting and location of several characteristics are included in the diabetic retinopathy (DR) classification. This takes a lot of time for doctors. Computers may gain classifications considerably faster after being trained, allowing them to aid clinicians in quick classification. Diabetic retinopathy is defined by morphological lesions in the retina that are related to abnormal retinal blood flow [12]. These lesions have a geographical distribution that can predict disease development and contain risk variables in the early stages of the disease.

This paper's contribution is completely exposed to the early identification of diabetic retinopathy (DR) by preprocessing the fundus retinal picture with the blood vessels separated. As deep learning models are able to extract crucial features from the input image automatically, we used a deep learning structure to segment the image to corroborate our guesses. To show the outcome, the preprocessed picture is fed into the trained CNN. The advantage of utilizing a trained CNN is that it can provide a faster diagnostic and report than an expert can. In diabetics, a yearly retinal examination and early identification of DR can significantly reduce the chance of visual loss.

## 2. Literature Review

The existence of lesions in the retina, which are produced by the illness, can help ophthalmologists forecast DR. Because of a lack of experience and equipment in some locations where diabetes is common and DR diagnosis and treatment is virtually always required, the suggested strategy is effective. The number of individuals suffering from diabetes is rising, and ophthalmologists are racing to avert blindness, yet DR infrastructure and professionals are in short supply. Gaussian smoothing, morphological top-hat filtering, and contrast enhancement are examples of image enhancement techniques. Enhancement is employed initially to boost contrast and minimize noise, and then adaptive local thresholding is utilized to perform the segmentation job [13]. Sundaram et al. suggested a hybrid segmentation strategy that employs methods such as morphology, multiscale vessel enhancement, and image fusion to emphasize blood vessels, that is, area-based morphology and thresholding [14]. Zhao et al. developed an infinite active contour model for autonomously segmenting retinal blood vessels, based on hybrid region information from the image for microscopic vascular structures [15]. Jiang et al. suggested a global thresholding-based morphological technique, in which capillaries are discovered through centerline detection, to find vessels quickly and correctly. Rodrigues et al. employed the wavelet transform and mathematical morphology to accomplish vascular segmentation, where tubular features of blood vessels were exploited to locate retinal veins and arteries [16]. To improve segmentation accuracy, Sazak et al. presented a retinal blood vessel image-enhancing approach. They employed the mathematical morphology patterns multiscale bowler-hat transform, in which vessel-like formations are recognized by thresholding after merging distinct structural elements [17].

Savelli et al. presented a new approach for segmenting vessels that compensated for lighting. To eliminate haze and shadow noise, a dehazing approach was utilized as a preprocessing approach, and classification was accomplished using a CNN trained on 800,000 patches with a dimension of 27 × 27 (the decision pixel was deemed the center pixel) [18]. Girard et al. created a fast machine learning strategy for segmenting vessels using a U-Net-inspired CNN for semantic segmentation, where the encoder and decoder provide down- and up-sampling of the image, accordingly. [19]. Hu et al. suggested a technique based on a CNN and conditional random fields (CRFs) for segmenting retinal vessels. This approach is divided into two phases: first, a multiscale CNN architecture with better cross-entropy loss function was used to the picture, and then CRFs were used to enhance the final output [20]. DeepVessel, a software that combines deep learning and CRFs, was presented by Fu et al. To learn rich hierarchical representations from pictures, a multiscale and multilevel CNN is employed [21]. Soomro et al. suggested a semantic segmentation network centered on deep learning and influenced by the well-known SegNet architecture. Grayscale data were created in the first phase using principal component analysis (PCA). The vessels were extracted. Semantic segmentation convolutional neural networks are used in the second step. After that, postprocessing was used to fine-tune the segmentation [22].

Jin et al. suggested a deep neural network based on a deformable U-Net. The network includes deformable convolutions, and an up-sampling operator is employed to improve the picture resolution and extract more accurate feature information [23]. Pixel CNN with batch normalization (PixelBNN), developed by Leopold et al., is centered on U-Net and pixel CNN and uses preprocessing to resize, decrease the dimension, and improve the picture [24]. Dense U-Net was employed as a semantic segmentation network for vascular segmentation by Wang et al. [25], with random transformations employed for data augmentation to increase the dense network's patch-based training effectiveness. For retinal vascular segmentation, Feng et al. suggested a cross-connected CNN (CcNet). Only the green channel of the fundus picture is used to train the CcNet; cross-connections and fusion of multiscale characteristics boost the network's performance [26]. Nevertheless, deep networks were employed in prior studies, which incorporated a large number of trainable parameters that boosted the network's complexity. To address these issues, this study offers a dual residual stream-based Vess-Net, which is not as deep as traditional semantic segmentation networks but provides good segmentation with a small number of trainable parameters and layers. The technique uses machine learning in the segmentation process to aid in the detection of retinopathy. Das et al. employed a CNN to train a diabetic retinopathy classifier and conduct classification. The CNN's classification structure is made up of a combination of squeeze and stimulation and bottleneck layers, one for each class, as well as a convolution and pooling layer architecture for classification between the two classes. When compared to standard systems, experimental findings suggest that the suggested method produces better outcomes. When tested on the DIARETDB1 data set [27], the model had an accuracy of 98.7% and a precision of 97.2%.

Shanthini et al. proposed a DR detection approach based on threshold segmentation. This approach used pixel-based segmentation to classify the foreground and background of the input retinal picture. A two-layer CNN is used to supplement the layer assessment process, which reduces false positives during classification. This procedure is followed in order to determine the exact detection of the retina's target region. Furthermore, the segment-based CNN (S-CNN) corrects the diagnostic fault using two hidden layers to distinguish between threshold and normalized circumstances based on categorization. The suggested technique is effective in improving detection accuracy, sensitivity, and true positives [28]. For the segmentation and localization of OD and fovea centers, Hasan et al. suggested the DRNet, an end-to-end encoder-decoder network. They suggested a skip link, called the residual skip connection, in the DRNet to compensate for the spatial information lost owing to encoder pooling. The suggested skip connection does not immediately concatenate low-level feature maps from the encoder's starting layers with the matching same scale decoder, unlike the U-Net's previous skip connection [29]. Other methods include genetic algorithm [30], two-path CNN [31], cascade CNN [32], patch shape selection method for feature extraction [33], FCM with mean-shift clustering method [34, 35], GARCH feature selection method [36], particle swarm algorithm for reducing surface roughness [37], and fatigue detection [38].

To identify and categorize DR from color fundus pictures, Jayanthi et al. utilized a novel particle swarm optimization (PSO) algorithm-based CNN model dubbed the PSO-CNN model. Preprocessing, feature extraction, and classification are the three steps of the proposed PSO-CNN algorithm. The PSO-CNN model is simulated using a benchmark DR database, and the experimental results show that the PSO-CNN model outperforms all other approaches by a substantial margin [39] (Table 1).

## 3. Methods and Materials

### 3.1. Fundus Photography

According to Singh et al. [5], fundus photography is a technique for photographing the back of the eye, which includes the retina, optic disc, and macula. Trained medical specialists can use fundus photography to observe and analyze the severity of the condition. For example, fundography pictures from DR-disease-selected data are shown in Figure 1.

### 3.2. Convolutional Neural Network

In this part, we will look into a convolutional neural network (CNN) model. One of the learning networks inspired by the perceptron neural net can be considered a neural network. This dynamic network has three layers: an input layer, an output layer, and a highly concealed layer. First, the problem's image or data are detected and put into the algorithm. The output layer's hidden weights would subsequently manifest themselves in a variety of ways [55–59]. A classification or recognition technique is used when the output has many numerical components, such as a binary number or index (e.g., image classification, normal = 1, and abnormal = 2). The findings are weighted after several photos have been trained. When a fresh picture, different than the training pictures, is introduced to the algorithm, the shape of the images is recognized. For example, if we train the computer with a matrix of diverse images, such as pictures of benign or malignant cancers, Alzheimer's, sarcoma, or brain tumors. Depending on the weights acquired, the approach indicates the type of disease. The CNN's base is the convolutional sublayer, and its output matrix is a three-dimensional neuron matrix. For a better understanding, typical neural networks are considered. In typical neural networks, each layer was nothing more than a list (one-dimensional as a rectangle) of neurons, each of which generated its own output and gradually amassed a sequence of outputs corresponding to each neuron. Instead of a single number, we are presented with a three-dimensional list (one cube) in which the neurons in the CNN are organized in three dimensions. As a consequence, this cube's output is a three-dimensional matrix as well [60, 61].

In traditional architecture, placing a pooling layer between multiple consecutive levels is a common approach. This layer seeks to minimize the number of variables and measurements in the grid, resulting in a reduced matrix (input) size by overfitting the display (width and height). The pooling layer works on each depth cut of the input matrix individually. The max-pooling option expands or contracts the size of the position. The activation process of artificial neural networks determines the node's output node or “neuron” based on the input or group of inputs. In the following node, this output is known as the input [62]. This occurs before a solution to the problem is identified. The results are transformed into a goal range, such as 0 to 1 or −1 to 1 (depending on the activation mechanism used). The logistic activation function, for example, transforms all inputs to true absolute ranges of 0 to 1. Optimizing your weight is another strategy to reduce weight. The rectified linear unit (ReLU) was used in this paper for the following functions [63]:

(1) $$\begin{array}{c} f\left(x\right)=\left\{\begin{array}{cc} 0 & x<0,\\ x & x\geq 0. \end{array}\right. \end{array}$$

Some activation functions, such as Softmax [49], are not limited to a single variable and may be applied to a vector or several variables employed in this paper:

(2) $$\begin{array}{c} f_{i}\left(\overset{⟶}{x}\right)=\frac{e^{x_{i}}}{\sum_{j=1}^{J}e^{x_{j}}}. \end{array}$$

A batch normalization layer is introduced to the network to normalize input data, speed up the training phase, and minimize network sensitivity between convolutional layers and nonlinearities. To create an aberrant image augmentation, a dropout layer on the fully connected layers is frequently utilized. We employed fully related layers at the end of the concealed layer, demonstrating to differentiate pictures. The output of the deep learning layer is a fully connected layer that guides the classification choice.

### 3.3. Receiver Operating Characteristic (ROC) Curve

The ROC curve is constructed by comparing the true-positive rate (TPR) to the false-positive rate (FPR) under various threshold conditions. The TPR is sometimes referred to as adaptability, recall, or likelihood of detection in machine learning. Starting on the left side of the ROC, we can observe that the FPR and TPR are both 0. (This suggests that the threshold line, which indicates the most test results, is long.) It is better to begin with the most test results and work your way up from there. The measurable and descriptive consistency of the outcomes of a measure separates knowledge into these two groups. The data may be split into positive and negative classes using sensitivity and attribute tests. The number of positive samples that can be adequately tested as positive is referred to as sensitivity. The number of negative examples that are correctly categorized as negative (positive = particular illness and negative = other cases) are referred to as specificity. The sensitivity of splitting the percentages of TP items into the number of true-positive and false-negative examples in mathematical terms [55, 64] is given as follows:

(3) $$\begin{array}{c} \text{sensitivity}=\frac{\text{TP}}{\text{TP}+\text{FN}}. \end{array}$$

The confusion matrix is the function of the approaches outlined in the field of artificial intelligence. This type of presentation is common in supervised learning algorithms, but it is also common in unsupervised learning. The expected value is shown in each column of the matrix. Assume that each row includes a valid (true) example. The name of this matrix is also given, allowing for mistakes and tampering with the result. This matrix is also characterized as a contingency matrix or an error matrix outside of artificial intelligence.

A machine learning classification model may be employed to predict the data point's actual class or its chance of belonging to multiple classes. The latter allows us to have more influence over the outcome. To understand the classifier's outcome, we may choose our own threshold. Depending on whether we want to reduce the number of false negatives or false positives, one of these criteria will almost certainly produce a better outcome than the others. The measurements alter when the threshold values vary. We may create a variety of confusion matrices and compare the results. It, however, would not be a wise decision. Alternatively, we can create a plot between some of these indicators so that we can quickly see which threshold is producing the best results.

The receiver operator characteristic (ROC) curve is a binary classification issue assessment measure. It is a probability curve that compares the TPR with the FPR at various threshold values, successfully distinguishing the signal from the noise. The area under the curve (AUC) is a summary of the ROC curve that measures a classifier's capability to discriminate between classes. The AUC indicates how well the model distinguishes between positive and negative classes. The higher the AUC number, the better. In a ROC curve, a higher *X*-axis value indicates that there are more false positives than true negatives. A higher *Y*-axis value indicates that there are more true positives than false negatives, whereas a lower *Y*-axis value indicates that there are fewer true positives. As a result, the threshold selection is based on the capacity to strike a balance between false positives and false negatives (Figure 2).

## 4. Results and Discussion

### 4.1. Data Collection

IDRiD (Indian Diabetic Retinopathy Image Dataset), the database used in this research, is the first of its kind to be representative of an Indian population. Furthermore, at the pixel level, this is the only data set that comprises both typical diabetic retinopathic lesions and normal retinal structures [61]. For each picture, this data set contains information on the severity of diabetic retinopathy and diabetic macular degeneration. This is appropriate for the creation and testing of image analysis algorithms for diabetic retinopathy early detection.

### 4.2. Blood Vessel Extraction Process

In this part, the suggested CNN for automated detection of DR was discussed. Figure 1 depicts the workflow of our suggested approach. First, the green channel preprocesses the input fundus retinal picture, and then CLAHE is utilized to improve the output from the green channel. The blood vessels are then extracted from the retinal fundus picture using multiple morphological techniques and binarization thresholding. Finally, the suggested CNN, which was constructed in MATLAB, is used to evaluate the segmented blood vessel in order to determine the severity of the DR automatically. Preprocessing methods are used to enhance the original image in order to increase the success rate of the planned task. Preprocessing procedures are used before segmenting blood vessels to ensure that the properties of the original picture are not altered. A preprocessing consists of five processes to eliminate these defects and provide more acceptable pictures for extracting the features: (1) green channel separation, (2) augmentation, (3) morphological procedures, (4) background subtraction, and (5) thresholding. Also, the histogram equalization approach generally improves the overall contrast of many pictures, primarily when a small number of intensity values represent the image. The intensities can also be better dispersed on the histogram with this modification, employing the whole range of intensities equitably. It enables locations with poor local contrast to get a boost in contrast. It is accomplished by histogram equalization, which effectively spreads out the densely packed intensity values that decrease picture contrast.  Figure 3 depicts a flow diagram for the segmentation of blood vessels procedure. The approaches are utilized to function well for the retinal pictures and are based on a trial-and-error method process. The following is a quick description of each step:

  Step 1: Green channel separation
  Because of red and blue channels of an RGB image suffer from noise and poor visual quality, the green channel is used to segment blood vessels. To increase the contrast of retinal images, the red and blue elements of the image are eliminated before processing. In the preprocessing step, the green channel is used to offer the best vasculature and contrast between the optic disc and the retinal tissue. As a consequence, the input image's green pixel values are extracted and saved as a vector.
  Step 2: Contrast enhancement
  Contrast-limited histogram equalization is a contrast enhancement technique that separates a big region into a number of little parts of similar size and works on each one separately to improve contrast. On the green channel, CLAHE is employed to help collect crucial blood vessel data. This method improves the quality of the image dynamically. It means that each part of the image is enhanced separately that causes no saturation in colors being observed. In Figure 4, the CLAHE is used to a fundus image.
  Step 3: Morphological processing
  The basic procedures of erosion and dilation are employed in mathematical morphology to investigate the relationship between a picture and a certain structuring element (SE). Dilation, erosion, opening, and closure are the most common procedures utilized here. This can be implemented by convolving (dot product) two sets of pixels, one of which contains the SE or kernel and the other of which contains the picture to be processed. Opening and closing are the two fundamental operators. Furthermore, dilation and erosion enlarge and reduce the size of an object inside the image, respectively. The SE, which is a matrix of just 0s and 1s with arbitrary size and form employed to examine the input picture, is a key element of these two procedures. The morphological opening and closing procedures are used to smooth the vessel's edge and the surrounding area, remove tiny holes, and fill in contour gaps. Algorithms combine the foregoing methods in the proposed work to recognize edges, eliminate noise and background, and discover specific forms in photos. There is not any problem when the input image has a different size, since the kernel size can be defined based on the size of aiming objects.
  Step 4: Background subtraction
  This strategy can be used to reduce anomalies in the backdrop of an image so that the foreground elements may be inspected more easily. The recommended method removes the backdrop by deleting some defined objects from the contrast-enhanced image.
  Step 5: Thresholding
  The practice of eliminating extraneous information from an image is known as thresholding. By eliminating all gray-level information from the fundus photographs, the blood vessels are converted to binary pixels. It is critical to distinguish between foreground blood vessels and background data. Thresholding is utilized to bring out hidden details as a result, selecting the appropriate threshold value is crucial, as a low number may reduce the size or amount of these items, whilst a high number may include extra background data. It is used to make a binary image with 1 (blood vessel) or 0 (background) pixel values so that numerical data may be read and fed into ML techniques.

### 4.3. Results of Segmentation Using the CNN Method

The findings of the CNN segmentation method are presented in this section. The detection method's architecture is depicted in Figure 5. It has 11 layers, including three convolutional layers. The input pictures are 256 × 256 grayscale fundus pictures taken from the eyes of DR patients, and the output layer includes ground truth from the IDRiD data set. The target tissue of the patient's eye is identified with 255 in these photos, whereas other spots are represented with zero values.

Colored pictures in the input picture in Figure 5 are converted to a dark-gray zone. It is difficult to recognize this area with the aid of a brain-computer. Given the possibility of deep learning approaches for segmenting regions with a broader range of hues than photographs with a similar color palette, more diverse colors have a better potential for segmentation. The target location is first discovered and labeled by medication or an automated method in this research. As a result, the target region's ground truth pictures are stored in the output layer of the proposed architecture. The presented architecture consists of 11 sublayers as shown in Table 2.

The segmentation results are depicted in Figure 6. The input picture of the DR eyes is shown in the first column of Figure 6. The second row, on the other hand, displays the ground truth image of the output layer. Seventy percent of pictures are utilized to train the network, and 30% are utilized to test the findings to begin the process. In the third column of Figure 6, the results of target region detection are displayed. We can see that the observations and the result are nearly identical. To improve the outcomes, all small regions from the findings are removed and replaced with a probability contour (fourth column). According to the findings, the suggested architecture is capable of detecting the target region with near-perfect accuracy. Figure 4 illustrates the training method.

Theoretically, the outcomes of segmentation algorithms are supplied with performance criteria. The ROC curve depicts the true-positive rate versus the false-positive rate. In the segmentation process, each image has its own set of criteria. Whether plots are shown with a higher true-positive rate and a smaller false-positive rate, data show that most photographs of ROC curves have an almost high performance (Figure 7(a)). To better understand the ROC curve using realistic figures, we provide the area under the curve (AUC) value. This criterion assesses whether values in the vicinity of one indicate high performance or not. In Figure 7(b), 92% of the images are in the high-performance range. This is something that can also be deduced from Figure 7(b). More than 90% of photographs are segmented accurately, with a 70% accuracy rate. At the completion of the process, the average amount of accuracy for all photographs is 83.84% (Figure 7(c)). The last requirement is the Jaccard value (Figure 7(d)), which depicts the overlapping regions of the generated image and ground facts. This number has ranged around 0.4 for many of the photos that have been produced. This lower score is due to the presence of black spots in the final photos when compared to ground truth data.

Table 3 compares the results of several techniques presented in the literature to standard incoherence evaluations. This approach achieves the best AUC and accuracy in terms of numbers but the minor sensitivity. This suggested approach obtains a mean sensitivity of 0.9% and accuracy of 83.8% in its overall performance.

## 5. Discussion

The most frequent way for ophthalmologists to diagnose DR is through a dilated eye examination. Fluorescein angiography, optical coherence tomography (OCT), and fundus photography are more ways to diagnose illness. The blood circulation and arterial anomalies are imaged during fluorescein angiography after an intravenous infusion of contrast dye. OCT is used to assess retinal anatomy, size, and edema (i.e., retinal swelling). Generally, DR diagnosis is arbitrary and requires a retina expert who has completed advanced training in diagnosis and grading. Visual evaluation and manual measurements of changes in retinal vasculature and layers are considered complicated duties. Regrettably, due to the lack of qualified eye-care experts and tertiary eye-care facilities, many diabetes patients seek to see a retina specialist only after they have symptomatic vision loss when their disease has progressed and is mainly permanent. As a result, an essential clinical motive is developing an objective and noninvasive diagnostic method to identify and evaluate DR properly at a preliminary phase.

CNNs have recently been used to diagnose diabetic retinopathy (DR) by evaluating fundus pictures, and their efficiency in segmentation and localization tasks has been demonstrated. DR is a severe consequence of diabetes that can lead to vision loss and possibly blindness. Such models provide good classification performance for the items in the training data set, but their use is limited to specialized areas such as DR detection. A broad range of complicated characteristics and their localizations within the picture is used to diagnose abnormal indications in fundoscopy. Each layer of CNN creates a new input image size by gradually extracting the most distinguishing features. Several approaches for improving accuracies, such as dimension reduction and feature augmentation, were presented in the state-of-the-art methods. Nonetheless, deep-learning-based DR detection research regularly indicates good performance in severe cases, whereas mild case detection remains difficult. Because of the probable absence of the early phase of DR, this restriction impedes the broader use of utterly automated mass-screening, perhaps leading to more complex condition future development.

A number of the study's flaws have been discovered. First, only small-to-moderate data set sizes were employed in the investigation because of the scarcity of DR pictures. To increase the data set, the necessary data augmentation techniques were used, such as rotation, horizontal/vertical flipping, and so on. Furthermore, when training the classifiers, the default hyperparameters were used. It was thought to be the most acceptable practice in the area. Nonetheless, tests with different optimizers were carried out. Lastly, the “black-box” aspect of deep-learning-based solutions is widely criticized, resulting in operator opposition to broader use.

## 6. Conclusion

The most prevalent cause of vision loss in diabetic patients is diabetic retinopathy. Other retinal and nonretinal visual issues, such as glaucoma, age-related macular degeneration, and neuropathy, can also cause visual deterioration or loss. Nonarterial optic ischemic neuropathy (NAION) and cataracts are examples of vascular vessels. Refractive errors, contrast sensitivity, direct light, and compliance amplitude should all be evaluated when a diabetic complains of visual problems. Physicians who treat diabetic patients utilize these vision issues to guarantee quick referral and treatment to prevent vision impairment, which can have a substantial impact on everyday living, especially for people who drive. Developing approaches that do not require the assistance of a doctor, even with smart technology such as phones, is critical. These procedures can also aid doctors in making an accurate and timely diagnosis of the condition. The investigation continues in the next section of the paper with the presentation of a segmentation approach for detecting target regions in human eyes. We devised a CNN architecture for pixel categorization of patients' eye fundus pictures in order to achieve our aim. For the output layer, we utilized preprocessed ground truth images. Seventy percent of the photos were utilized for training data, with the remaining photos being utilized to validate the provided architecture. The provided approach can practically recognize the target region of eye pictures with high accuracy of 83.84%, according to the results. This network may also be used to treat patients better by separating the target region from their eye pictures. It is past time for artificial intelligence to be used in medicine to assist doctors in making better and faster diagnoses.

## Figures and Tables

**Figure 1:** Different classes of disorders in DR disease [24]: (a) original image, (b) microaneurysms, (c) haemorrhages, (d) hard exudates, (e) soft exudates, and (f) optic disc.

**Figure 2:** The ROC curve sample.

**Figure 3:** The process of blood vessel extraction from fundus images.

**Figure 4:** The training process of the CNN approach.

**Figure 5:** The architecture of the CNN method for segmentation of fundus images.

**Figure 6:** Examples of segmentation of fundus images of DR patients.

**Figure 7:** Results of segmentation: (a) ROC cure, (b) AUC criteria, (c) accuracy of segmentation, and (d) Jaccard criteria.

**Table 1:** Literature review of DR images segmentation.

Methods	Strength	Weakness
Vessel segmentation using thresholding [40–42]	Approximation of vessel pixels using a simple approach	When the vessel pixel values are closer to the background, false points are recognized
Fuzzy-based segmentation [43]	With consistent pixel values, it works great	To increase the responsiveness of blood vessels, extensive preprocessing is necessary
Active contours [44]	For detection of real boundaries, a better approximation is used	Processes that are iterative and time-consuming are necessary
Vessel tubular properties-based method [16]	Approximation of vessel-like structures is excellent	Pixel discontinuities put restrictions on how far you can go
Line detection-based method [45]	The removal of the backdrop aids in the reduction of fake skin-like pixels	
Random forest classifier-based method [46]	To identify pixels, use a lighter technique	Before categorization, many transformations are required to produce features
Patch-based CNN [47]	Better categorization	Training and testing take a long time to complete
SVM-based method [48]	Training time is reduced	To create a feature vector, preprocessing approaches involving many photos are used
Extreme machine learning [49]	Machine learning has a lot of differentiating factors	To create distinguishable features, morphology and other traditional procedures are required
Mahalanobis distance classifier [49]	Training is a simple operation	To compute relevant features, preprocessing overhead is still necessary
U-Net-based CNN for semantic segmentation [19]	The boundaries are nicely preserved by the U-Net construction	Preprocessing in gray scale is necessary
Multiscale CNN [20]	Multireceptive fields improve learning	In other circumstances, tiny vessels are not recognized
CNN with CRFs [20]	Faster segmentation is achieved using a CNN with a few layers	CRFs are difficult to compute
SegNet-inspired method [22]	The design of encoders and decoders creates a unified network layer topology	PCA is used to prepare data for training purposes
CNN with visual codebook [50]	For correlation with ground truth representation, a 10-layer CNN is used	There is no end-to-end training and testing mechanism
CNN with quantization and pruning [51]	Convolutions that have been pruned improve the network's efficiency	The number of trainable parameters increase as layers are fully coupled
Three-stage CNN-based deep learning method [52]	A compelling representation is provided by the fusion of multifeature images	The use of three CNNs necessitates a higher level of computing power and expense
Modified U-Net with dice loss [53]	Dice loss provides good results with unbalanced classes	PCA is used to prepare data for training purposes
Deformable U-Net-based method [23]	When classes are unequal, dice loss delivers acceptable results	Patch-based training and testing take a lot of time
PixelBNN [24]	Pixel is a term that refers to CNN is well-known for its ability to forecast pixels with spatial dimensions	CLAHE is used for preprocessing
Dense U-Net-based method [25]	The use of a dense block can help solve the problem of disappearing gradients	Patch-based training and testing take a lot of time
Cross-connected CNN (CcNet) [26]	Layer cross-connections provide features more power	Preprocessing is used to create a complex architecture
Vess-Net [54]	With fewer layers, robust segmentation is possible	To properly train the network, augmented data is required

**Table 2:** The architecture of presented CNN layers.

No.	Layer name	Properties
1	Image input	256 × 256 × 1 images with “zerocenter” normalization
2	Convolution	32 (3 × 3 × 1) convolutions with stride [1 1] and padding [1 1 1 1]
3	ReLU	
4	Dropout	50% dropout
5	Max pooling	2×2 max pooling with stride [2 2] and padding [0 0 0 0]
6	Convolution	64 (3 × 3 × 32) convolutions with stride [1 1] and padding [1 1 1 1]
7	ReLU	
8	Transposed convolution	32 (4 × 4 × 64) transposed convolutions with stride [2 2] and cropping [1 1 1 1]
9	Convolution	2 (1 × 1 × 32) convolutions with stride [1 1] and padding [0 0 0 0]
10	Softmax	
11	Pixel classification	Dice loss

**Table 3:** Comparison between presented methods and the state-of-the-art methods.

Authors	Method	Sensitivity	Accuracy
Li et al. [65]	Cross-modality method	0.757	0.953
Christodoulidis et al. [66]	Multiscale tensor voting	0.851	0.948
Aslani and Sarnel [67]	Multiscale Gabor wavelet	0.755	0.951
Vega et al. [68]	Lattice neural networks	0.744	0.941
Jebaseeli et al. [69]	Average value	0.806	0.995
Presented method	CNN	0.891	0.838

## Data Availability

The data set IDRiD (Indian Diabetic Retinopathy Image Dataset) is available online at https://ieee-dataport.org/open-access/indian-diabetic-retinopathy-image-dataset-idrid.
